# Long Noncoding RNA OIP5-AS1 Promotes the Disease Progression in Nasopharyngeal Carcinoma by Targeting miR-203

**DOI:** 10.1155/2021/9850928

**Published:** 2021-02-05

**Authors:** Jian Tang, Chengxiao Fu, Yanwen Li, Shuangqin Chen, Xiaoxin Jiang, Wenqian Xu, Haitao Xie

**Affiliations:** ^1^Department of Infectious Disease, The First Affiliated Hospital, University of South China, Hengyang 421001, China; ^2^Department of Pharmacy, The First Affiliated Hospital, University of South China, Hengyang 421001, China; ^3^Department of Laboratory Medicine, The First Affiliated Hospital, University of South China, Hengyang 421001, China; ^4^Department of Neurology, The First Affiliated Hospital, University of South China, Hengyang 421001, China

## Abstract

Nasopharyngeal carcinoma (NPC) is a kind of malignancy generated from the nasopharyngeal epithelium. Recently, long noncoding RNA (lncRNA) has been shown to be involved in the regulation of many signaling pathways and is closely associated with carcinogenesis and tumor progression. However, the precise role of lncRNA Opa-interacting protein 5 antisense RNA 1 (OIP5-AS1) in NPC is not well understood. Here, we find that OIP5-AS1 is overexpressed in NPC patient specimens and NPC cell lines. Further investigations reveal that knockdown of OIP5-AS1 significantly inhibits the proliferation, migration, and invasion and accelerates the apoptosis of NPC cells *in vitro.* Consistent with these findings, NPC progression is significantly slowed in mice when OIP5-AS1 is knocked down. Interestingly, there is a functional link between OIP5-AS1 and microRNA-203 (miR-203), a tumor suppressor, in NPC cells. In conclusion, our data demonstrate that OIP5-AS1 plays an important role in the development and progression of NPC by targeting miR-203 and therefore provide a promising target for the treatment of NPC.

## 1. Introduction

Nasopharyngeal carcinoma (NPC) is a malignancy of the epithelium located in the nasopharynx, which is very common in South China and Southeast Asia, presenting a distinct geographical distribution in occurrence [1]. It is known that there are three main factors, including genetic susceptibility, Epstein-Barr virus infection, and environmental factors, which could cause NPC [2]. A large amount of NPC patients are diagnosed at an advanced stage due to the special anatomical location and inconspicuous early symptoms [3]. At present, radiation therapy alone or in combination with chemotherapy is widely used to treat NPC [4]. Although the overall survival rate is gradually improved, the side effects of these strategies seriously affect the life quality of NPC patients [5]. Therefore, it is important to deeply explore the biological mechanism and find new therapeutic targets for NPC.

During the transcription and translation of genetic information, about 98.5% of the RNAs do not have the ability to be translated into proteins [6, 7]. Long noncoding RNA (lncRNA) is one of these types of RNAs, with a length greater than 200 nucleotides [8, 9]. Accumulating evidence suggests that lncRNA plays an important role in regulating various physiological or pathological processes by interacting with cellular macromolecules, including DNA, RNA, and protein [10]. Although several lncRNAs, such as ANRIL, NEAT1, and HOTAIR, have been recognized to be implicated in the pathogenesis of nasopharyngeal carcinoma [11–13], the underlying mechanisms have not been completely uncovered.

Opa-interacting protein 5 antisense RNA 1 (OIP5-AS1) is a newly recognized lncRNA that is located on the opposite strand of the human OIP5 gene [14]. Recently, studies reported that OIP5-AS1 plays a tumor-promoting role in multiple types of cancers, such as hepatocellular carcinoma, lung cancer, and oral squamous cell carcinoma [15–17]. Of note, OIP5-AS1 promotes the development and progression of these cancers through modulation of different pathways, which is in line with the notion that the function of lncRNA is highly heterogeneous in different tissues [18]. However, the specific role and mechanism of OIP5-AS1 in NPC have not been illustrated.

In this study, we first observed that OIP5-AS1 expression level was significantly upregulated in nasopharyngeal carcinoma tissues compared to normal tissues. In addition, the upregulation of OIP5-AS1 was associated with poor prognosis in patients with nasopharyngeal carcinoma. Further research showed that OIP5-AS1 facilitated the progression of nasopharyngeal carcinoma via negative regulation of miR-203. Overall, our data indicate that OIP5-AS1 plays a carcinogenic role in NPC and may be a potential therapeutic target.

## 2. Materials and Methods

### 2.1. General Materials

A total of 105 NPC patients who underwent biopsy in our hospital from 2011 to 2015 were enrolled in this study. Clinical NPC tissues and adjacent normal tissues were collected and then confirmed by pathological examination. Neither the radiotherapy and chemotherapy nor targeted drugs were given to any patients before operation. All tissues were immediately placed in liquid nitrogen in a freezing tube following surgery and then stored at -80°C until further experiments. All patients have signed the written informed consent form. This study was authorized by the Ethics Committee (the First Affiliated Hospital of South China University).

### 2.2. Cell Culture

Nasopharyngeal epithelial cells NP69 and human NPC cell lines (C666-1, 5-8F, HNE-1, S18, CNE-1, and CNE-2) were obtained from the Cell Bank of the Chinese Academy of Sciences (Shanghai, China) and then routinely grown in RPMI-1640 medium (Gibco, Carlsbad, CA, USA) containing 10% fetal bovine serum (FBS; Gibco) and 100 U/ml penicillin/streptomycin (Life Technologies, USA). All cells were kept in a humidified atmosphere with 5% CO_2_ at 37°C.

### 2.3. Lentivirus Transduction and Cell Transfection

The lentivirus expressing small hairpin RNA sh-OIP5-AS1 or negative control (sh-NC) was obtained from Hanbio Co., Ltd. (Shanghai, China) and then transduced into NPC cell lines using polybrene (Hanbio Co., Ltd.). miR-203-inhibitor or negative control (GenePharma Co., Ltd., Shanghai, China) was transfected into cells using Lipofectamine 3000 (Invitrogen, Carlsbad, CA, USA) following the manufacturer's instructions. The sequence of sh-OIP5-AS1 is as follows: 5′-CAAACAGGCUUUGUGUUCCUUAUCA-3′.

### 2.4. Quantitative RT-PCR (qRT-PCR)

Total RNA was extracted from samples using the RNAiso Plus reagent (Takara Biotechnology Co., Ltd., Dalian). Then, 1 *μ*g of RNA was converted to cDNA using the PrimeScript RT kit (Takara, Tokyo, Japan). After that, gene expression was quantified by qRT-PCR using the SYBR PremixEx Taq™ II kit (Takara) and standardized to GAPDH. Primer sequences are as follows: OIP5-AS1, forward 5′-GGTCGTGAAACACCGTCG-3′ and reverse 5′-GTGGGGCATCCAGGGT-3, and GAPDH, forward 5′-TGTTCGTCATGGGTGTGAAC-3′ and reverse 5′-ATGGCATGGACTGTGGTCAT-3′. The expression of miRNAs was measured using the mirVana qRT-PCR miRNA Detection kit (Invitrogen). The primers of miRNAs were purchased from Guangzhou RiboBio Co., Ltd. (China). Small RNA U6 was used as an internal reference gene. The following primers were used: miR-203, forward 5′-CGATGCTGTGAAATGTTTAGGGAC-3′ and reverse 5′-TATGGTTTTGACGACTGTGTGAT-3′; miR-342-3p, forward 5′-AGGAGTCTCACACAGAAATCGCA-3′ and reverse 5′-GTGCAGGGTCCGAGGT-3′; miR-422a, forward 5′-AAGCACTGGACTTAGGGTCA-3′ and reverse 5′-GTGCAGGGTCCGAGGT-3′; miR-204-5p, forward 5′-ACACTCCAGCTGGGTTCCCTTTGTCATCCTAT-3′ and reverse 5′-CTCAACTGGTGTCGTGGA-3′; and U6 snRNA, forward 5′-ATTGGAACGATACAGAGAAGATT-3′ and reverse 5′-GGAACGCTTCACGAATTTG-3′.

### 2.5. Western Blotting

Total proteins were extracted with RIPA Lysis (Thermo Fisher Scientific) and then separated by 10% of SDS-PAGE and transferred into the PVDF membranes (Millipore, Billerica, MA, United States). After blocking with bovine serum albumin (Sigma-Aldrich, St. Louis, MO, United States) for 1 hour at 37°C, the membranes were incubated with primary antibodies: cleaved (Cle) caspase-3 (Abcam, Cambridge, UK), caspase-3 (Abcam), cleaved (Cle) caspase-9 (Cell Signaling Technology, Danvers, MA, USA), caspase-9 (Cell Signaling Technology), ZEB2 (Abcam), E2F3 (Abcam), CDH6 (Abcam), and GAPDH (Abcam) at 4°C overnight. Subsequently, the membranes were incubated with the secondary antibodies and measured with the ECL Chemiluminescence Detection System (Thermo Fisher Scientific, Rochester, New York).

### 2.6. Colony Formation and Cell Proliferation Assays

For the colony formation assay, 5 × 10^3^ cells were seeded into 6-well plates and incubated in RPMI-1640 containing 10% FBS for 14 days. Subsequently, cells were fixed with 4% paraformaldehyde and stained with 0.1% crystal violet (Beyotime, Shanghai, China) for 30 min. The number of colonies containing more than 50 cells was counted. For the cell proliferation assay, cells were plated into 96-well plates at a density of 3 × 10^3^/well. At indicated time (24-96 hours) after culture, 10 *μ*l of Cell Counting Kit-8 solution (CCK-8; Dojindo, Kumamoto, Japan) was added into each well. After culturing for another 2 hours at 37°C, the samples were detected by using a microplate reader (Thermo Fisher Scientific, Waltham, MA) set at 450 nm.

### 2.7. Cell Invasion and Migration Assays

Cell invasion and migration assays were performed using the Transwell Matrigel Chambers (8 *μ*m pore size; Corning, Beijing, China) as described previously [15]. The number of invaded or migrated cells was counted using a microscope.

### 2.8. Flow Cytometric Analysis

For cell cycle analysis, cells were collected and fixed in 70% ethanol overnight. After being washed in phosphate-buffered saline (PBS) and digested with RNase A, cells were stained with propidium iodide (PI), followed by flow cytometric analysis. Cells apoptosis was detected using the Annexin V-APC/7-AAD kit (BioLegend, San Diego, CA, USA) following the manufacturer's instructions. The samples were measured on a FACSCanto (BD Biosciences, San Diego, CA, USA) flow cytometer and analyzed using the FlowJo 10.0 software (TreeStar, San Carlos, CA, USA).

### 2.9. Luciferase Reporter Assay

The wild-type or mutant OIP5-AS1 synthesized from Sangon Biotech (Shanghai, China) were cloned into a psiCHECK-2 vector (Promega Biotech Co., Ltd., Madison, Wisconsin, USA). Then, these vectors, together with miR-203 mimic or control obtained from GenePharma Co., Ltd., were cotransfected into 293T cells using Lipofectamine 3000 (Invitrogen). The luciferase activity was measured using the Dual-Luciferase Reporter Assay Kit (Promega Biotech Co., Ltd.) after being transfected for 48 hours. Renilla luciferase was used as an internal reference.

### 2.10. Animal Experiments

BALB/C nude mice (male, 5-6 weeks old, weighing 18 ± 2 g) were purchased from Beijing Biocytogen Co., Ltd. (China) and housed in a specific pathogen-free environment at 22-24°C with a regular 12-hour day/night cycle. And then, 1 × 10^7^ cells infected with or without sh-OIP5-AS1 were subcutaneously injected into the mice. Tumor volume was measured with a caliper every one week. At 5 weeks after implantation, all mice were euthanized and tumor tissues were excised for weight evaluation and other experiments. This study was authorized by the Animal Care and Use Committee (the First Affiliated Hospital of South China University).

### 2.11. Statistical Analysis

All experiments were repeated for three times independently. Student's *t*-test was used to compare the difference between two groups, and one-way ANOVA was used to compare the difference among multiple groups. Statistical data analysis was carried out using GraphPad Prism 6.0 (GraphPad Software, Inc., La Jolla, CA) statistical packages. Results were shown as the mean ± standard deviation (SD). ^∗^*p* < 0.05 was defined as statistically significant.

## 3. Results

### 3.1. OIP5-AS1 Is Overexpressed in NPC Specimens and Cell Lines

In order to explore the role of OIP5-AS1 in the development and progression of NPC, 105 cases of NPC specimens and adjacent noncancerous nasopharyngeal tissues were collected. Then, qRT-PCR analysis revealed that OIP5-AS1 expression was highly increased in NPC tissues compared with the corresponding controls (Figure 1(a)). In addition, the level of OIP5-AS1 was significantly higher in several NPC cell lines than in the nasopharyngeal epithelium cell NP69 (Figure 1(b)). Based on the finding that OIP5-AS1 was much higher in 5-8F and CNE-1 cells, these cells were chosen to conduct the following experiments. On the other hand, NPC patients were divided into a high group and a low group according to the median of OIP5-AS1 expression. Interestingly, the Kaplan-Meier survival analysis showed that NPC patients with low OIP5-AS1 expression had longer survival times (Figure 1(c)). These results suggest that OIP5-AS1 may be involved in the pathogenesis of NPC.

### 3.2. Knockdown of OIP5-AS1 Inhibits the Proliferation of NPC Cells

To determine whether OIP5-AS1 contributes to the malignant phenotype of NPC, we knocked down OIP5-AS1 expression in 5-8F and CNE-1 cells through lentiviral transduction (Figure 2(a)). It was found that knockdown of OIP5-AS1 significantly decreased colony formation and proliferation of NPC cells *in vitro* (Figures 2(b) and 2(c)). Moreover, cell cycle progression was also inhibited in NPC cells after knockdown of OIP5-AS1 by flow cytometric analysis (Figure 2(d)). These data indicate that OIP5-AS1 may control the proliferation of NPC cells.

### 3.3. Knockdown of OIP5-AS1 Accelerates the Apoptosis and Decreases the Migration and Invasion of NPC Cells

We next evaluated whether knockdown of OIP5-AS1 also affects NPC cell apoptosis. Flow cytometric analysis displayed that decreasing OIP5-AS1 expression significantly accelerated the apoptosis of NPC cells (Figures 3(a)–3(d)). Meanwhile, several proapoptotic proteins (including cleaved caspase-3 and cleaved caspase-9) were upregulated in NPC cells after OIP5-AS1 knockdown by western blot analysis (Figure 3(d)). On the other hand, using Transwell assays, we found that knockdown of OIP5-AS1 suppressed the migration and invasion of NPC cells (Figures 3(e)–3(h)), hinting that OIP5-AS1 may be involved in NPC cell metastasis.

### 3.4. Knockdown of OIP5-AS1 Accelerates NPC Growth *In Vivo*

To further confirm whether knockdown of OIP5-AS1 affects the tumorigenesis ability of NPC cells *in vivo*, we subcutaneously injected sh-NC- or sh-OIP5-AS1-transfected 5-8F cells into BALB/c nude mice. Consistent with the in vitro observations, the tumor volume formed in the sh-OIP5-AS1 group was substantially smaller than that in the sh-NC group (Figures 4(a) and 4(b)). Meanwhile, the tumor weight was also distinctly lower in the sh-OIP5-AS1 group than in the sh-NC group 35 days after implantation (Figure 4(c)). Then, the downregulated expression of OIP5-AS1 in the tumor xenografts formed by sh-OIP5-AS1-transfected 5-8F cells was also determined using qRT-PCR (Figure 4(d)). Collectively, our data suggest that OIP5-AS1 plays an important role in NPC growth *in vivo*.

### 3.5. OIP5-AS1 Directly Binds to miR-203 and Suppresses Its Expression

Accumulating evidences have shown that lncRNA can serve as a sponge to bind to specific miRNAs; we therefore hypothesized that OIP5-AS1 could inhibit some antitumor miRNAs in NPC cells. Bioinformatics analysis using starBase v3.0 (http://www.sysu.edu.cn) revealed that some previously recognized antitumor miRNAs have a potential binding site in OIP5-AS1, including miR-342-3p, miR-422a, miR-204-5p, and miR-203 [19–22]. Interestingly, we observed that only miR-203 was significantly increased in NPC cells after OIP5-AS1 knockdown (Figure 5(a)). Meanwhile, the expression of miR-203 was lower in NPC tissues than in normal tissues (Figure 5(b)), which was consistent with a previous study [23]. Similarly, the expression of miR-203 was also significantly downregulated in NPC cell lines (Figure 5(c)). More importantly, miR-203 expression was negatively correlated with the level of OIP5-AS1 in NPC tissues (Figure 5(d)). In addition, several miR-203 target genes (including ZEB2, E2F3, and CDH6), known to aggravate the NPC phenotype [23–25], were downregulated in NPC cells when OIP5-AS1 was knocked down (Figures 5(e) and 5(f)). To further verify this concept, we performed the luciferase reporter gene assay and found that OIP5-AS1 can directly bind to miR-203 (Figure 5(g)). Therefore, our data illuminate that OIP5-AS1 modulates NPC progression probably via sponging miR-203.

### 3.6. OIP5-AS1/miR-203 Axis Modulates NPC Progression

Finally, we tried to prove whether OIP5-AS1 promotes the progression of NPC by inhibiting the expression of miR-203. In fact, we noticed that the inhibition of miR-203 using a miR-203-inhibitor significantly recovered the proliferation, colony formation, cell cycle, migration, and invasion and reduced the apoptosis of NPC cells with OIP5-AS1 knockdown (Figures 6(a)–6(g)). Furthermore, miR-203 suppression also markedly increased the expression of ZEB2, E2F3, and CDH6 in OIP5-AS1-knockdown NPC cells (Figures 6(h) and 6(i)). Taken together, our findings demonstrate that the OIP5-AS1/miR-203 axis plays a critical role in modulating the pathogenesis of NPC.

## 4. Discussion

Nasopharyngeal carcinoma is the most common malignancy in the neck and head [26]. Despite the advances in diagnostic and therapeutic strategies, the prognosis of this disease is not very satisfactory due to the high relapse and distant metastasis [27]. Therefore, a deep understanding of molecular mechanisms underlying the development and the progression of NPC is needed. In this study, we report for the first that OIP5-AS1 function as an oncogene and play a critical role in NPC development and progression by targeting miR-203.

Many studies have implicated that lncRNA participates in many biological processes and that the abnormal expression of lncRNA is closely related to the occurrence and development of a variety of human diseases, including cancers [9, 28, 29]. However, because of the diversity of species and heterogeneity of functions, many lncRNAs have not been thoroughly investigated. It has been reported that lncRNA OIP5-AS1 is involved in regulating the pathogenesis of several cancers. For instance, OIP5-AS1 increases SOX4 expression to induce hepatocellular carcinoma through sponging miR-363-3p [15]. Meantime, OIP5-AS1 affects oral squamous cell carcinoma progression via modulating miR-338-3p and targeting NRP [17]. However, its role in NPC has not been explored. In the present study, we observed that the OIP5-AS1 was overexpressed in NPC samples obtained from patients with NPC and NPC patients with high expression of OIP5-AS1 had a lower survival rate, suggesting that OIP5-AS1 may regulate the biology of NPC.

It has been well established that cancer cells are characterized by uncontrolled cell proliferation and decreased apoptosis [30, 31]. In this research, we found that OIP5-AS1 knockdown significantly suppressed the colony formation, proliferation, and cell cycle progression *in vitro*. In addition, decreasing OIP5-AS1 expression evidently increased the apoptosis of NPC cells, accompanied by the upregulation of several critical proapoptotic proteins. On the other hand, early lymph node metastasis is common in NPC patients [32]. Indeed, Transwell assays showed that knockdown of OIP5-AS1 suppressed the migration and invasion of NPC cells. In accordance with these findings, knockdown of OIP5-AS1 slowed the growth of tumors in nude mice. Therefore, our results indicate that OIP5-AS1 is a critical protooncogene in NPC.

miRNA is a kind of small non-protein-coding RNA with a length of 21-24 bases [33]. As we know, miRNAs are widely involved in regulating cell behaviors mainly through degrading target mRNA or inhibiting the translation of the target gene [34]. In recent years, the function of miRNA in tumor cells has been widely publicized. It is crucial that lncRNA, as an endogenous competitive RNA, can specifically bind to miRNAs and regulate their expression [35]. In our study, we observed that knockdown of OIP5-AS1 led to a marked increase in miR-203 expression in NPC cells. In fact, miR-203 is an important tumor suppressor in NPC or other tumor cells [36, 37]. It was reported that miR-203 can restrain the proliferation and metastasis and promotes the apoptosis of cancer cells [38, 39], which is consistent with our results. Further investigations displayed that there was a negative relationship between OIP5-AS1 and miR-203 in NPC tissues. In addition, the miR-203 target genes (ZEB2, E2F3, and CDH6) that have been reported to promote NPC progression were evidently decreased in NPC cells after OIP5-AS1 knockdown. Specifically, the luciferase reporter assay confirmed that OIP5-AS1 can sponge miR-203 and inhibit its expression. Finally, inhibiting the expression of miR-203 significantly recovered the proliferation, cell cycle, colony formation, invasion, and migration and reduced the apoptosis in OIP5-AS1-knockdown NPC cells. These results proved that OIP5-AS1 promotes the progression of NPC, at least in part, by inhibiting miR-203. On the one hand, considering that, lncRNA can regulate cell biological function in a variety of ways [40, 41]. Therefore, we cannot deny that there may be other mechanisms which also mediate partial function of OIP5-AS1 on NPC.

In summary, the findings presented in this study suggest that OIP5-AS1 play an oncogenic role in NPC by negatively modulating the tumor suppressor miR-203. Therefore, this study further reveals the underlying mechanism of NPC development and progression and provides a new target for the treatment of NPC.

## Figures and Tables

**Figure 1:** OIP5-AS1 is overexpressed in NPC specimens and cell lines. (a) The relative expression of OIP5-AS1 in NPC specimens and adjacent tissues obtained from 105 patients, determined by qRT-PCR. (b) The expression of OIP5-AS1 in NPC cell lines (C666-1, 5-8F, HNE-1, S18, CNE-1, and CNE-2) and the nasopharyngeal epithelium cell NP69, determined by qRT-PCR. (c) The overall survival of NPC patients with high or low OIP5-AS1 expression (based on the median expression levels). ^∗^*p* < 0.05, ^∗∗^*p* < 0.01.

**Figure 2:** Knockdown of OIP5-AS1 inhibits the proliferation of NPC cells. (a) qRT-PCR analysis of the expression of OIP5-AS1 in 5-8F and CNE-1 cells with or without knockdown of OIP5-AS1. (b) The colony formation of 5-8F and CNE-1 cells with or without knockdown of OIP5-AS1. (c) The proliferation of 5-8F and CNE-1 cells with or without knockdown of OIP5-AS1, determined by the CCK-8 assay. (d) Cell cycle analysis of 5-8F and CNE-1 cells with or without knockdown of OIP5-AS1, detected by flow cytometry. ^∗∗^*p* < 0.01.

**Figure 3:** Knockdown of OIP5-AS1 accelerates the apoptosis and decreases the migration and invasion of NPC cells. (a, b) The apoptosis of 5-8F and CNE-1 cells with or without knockdown of OIP5-AS1, detected by flow cytometry. (c, d) Western blot analysis of the expression of apoptosis-associated proteins in 5-8F and CNE-1 cells with or without knockdown of OIP5-AS1. Relative expression of cleaved (Cle) caspase-3 and cleaved (Cle) caspase-9 was normalized to caspase-3 and caspase-9, respectively. (e–h) Transwell assay showing the cell (e, f) migration and (g, h) invasion of 5-8F and CNE-1 cells with or without knockdown of OIP5-AS1. ^∗∗^*p* < 0.01.

**Figure 4:** Knockdown of OIP5-AS1 accelerates NPC growth *in vivo*. (a–d) BALB/c nude mice were subcutaneously injected with 5-8F cells transfected with sh-NC or sh-OIP5-AS1. (a) Tumor volume was measured once every 7 days. (b, c) Five weeks after implantation, all mice were sacrificed, and then, tumor tissues were collected and weighed. (d) Meanwhile, OIP5-AS1 expression in tumor tissues was detected by qRT-PCR. ^∗∗^*p* < 0.01.

**Figure 5:** OIP5-AS1 directly binds to miR-203 and suppresses miR-203 expression. (a) The relative expression of miR-342-3p, miR-422a, miR-204-5p, and miR-203 in 5-8F and CNE-1 cells after knockdown of OIP5-AS1. (b) The relative expression of miR-203 in NPC tissues and adjacent normal tissues obtained from 105 patients. (c) The relative expression of miR-203 in NPC line cells and the nasopharyngeal epithelium cell NP69. (d) Pearson correlation analysis revealing a significantly negative relationship between miR-203 and OIP5-AS1 in NPC patient specimens (*r* = −0.5752, *p* < 0.01). (e, f) Western blot analysis of the expression of ZEB2, E2F3, and CDH6 in 5-8F and CNE-1 cells with or without knockdown of OIP5-AS1. Relative expression of ZEB2, E2F3, and CDH6 was normalized to GAPDH. (g) starBase 3.0 analysis revealing the specific binding site of miR-203 in OIP5-AS1. Relative luciferase activity in 293T cells after cotransfected with OIP5-AS1 (WT or MUT) and miR-203 mimic (or miR-NC). WT: wild type; MUT: mutant type; NC: negative control. ^∗^*p* < 0.05, ^∗∗^*p* < 0.01.

**Figure 6:** The OIP5-AS1/miR-203 axis modulates NPC progression. (a–i) OIP5-AS1-knockdown 5-8F and CNE-1 cells were treated with miR-inhibitor-NC or miR-203-inhibitor. After that, (a) the expression of miR-203 was measured by qRT-PCR. And then, the (b) proliferation, (c) colony number, (d) cell cycle, (e) apoptosis, (f) migration, and (g) invasion were determined. Finally, (h, i) the expression of ZEB2, E2F3, and CDH6 was detected by western blot. Relative expression of ZEB2, E2F3, and CDH6 was normalized to GAPDH. ^∗∗^*p* < 0.01.

## Data Availability

The dataset supporting the conclusions of this article is included within the article.
